The article "A three-dimensional (3-D) meshfree-based computational model to investigate stress-strain-time relationships of plant cells during drying" was published in 2020. Journal: PLoS One.

# A three-dimensional (3-D) meshfree-based computational model to investigate stress-strain-time relationships of plant cells during drying

**DOI:** 10.1371/journal.pone.0235712

**Published:** 2020-07-07

**Authors:** C. M. Rathnayaka, H. C. P. Karunasena, W. D. C. C. Wijerathne, W. Senadeera, Y. T. Gu

**Affiliations:** 1 Science and Engineering Faculty, School of Mechanical, Medical and Process Engineering, Queensland University of Technology (QUT), Brisbane, Australia; 2 Department of Mechanical and Manufacturing Engineering, Faculty of Engineering, University of Ruhuna, Galle, Sri Lanka; 3 Department of Science and Technology, Faculty of Applied Sciences, Uva Wellassa University, Badulla, Sri Lanka; 4 School of Mechanical and Electrical Engineering, University of Southern Queensland, Springfield, Australia; University of New South Wales, AUSTRALIA

## Abstract

A better understanding of plant cell micromechanics would enhance the current opinion on “*how things are happening*” inside a plant cell, enabling more detailed insights into plant physiology as well as processing plant biomaterials. However, with the contemporary laboratory equipment, the experimental investigation of cell micromechanics has been a challenging task due to diminutive spatial and time scales involved. In this investigation, a three-dimensional (3-D) coupled Smoothed Particle Hydrodynamics (SPH) and Coarse-Grained (CG) computational approach has been employed to model micromechanics of single plant cells going through drying or dehydration. This meshfree-based computational model has conclusively demonstrated that it can effectively simulate the behaviour of stress and strain in a plant cell being compressed at different levels of dryness: ranging from a fresh state to an extremely dried state. In addition, different biological and physical circumstances have been approximated through the proposed novel computational framework in the form of different turgor pressures, strain rates, mechanical properties and cell sizes. The proposed computational framework has potential not only to study the micromechanical characteristics of plant cellular structure during drying, but also other equivalent, biological structures and processes with relevant modifications. There are no underlying difficulties in adopting the model to replicate other types of cells and more sophisticated micromechanical phenomena of the cells under different external loading conditions.

## Introduction

Plant materials are comprised of biological tissues, where each tissue is approximated as a network of plant cells separated by intercellular spaces. Water plays a key role in facilitating biological activities inside the tissue, and a plant cell usually stores more than 90% of water by its mass in the vacuoles and cell walls [1]. Whenever a water potential gradient is generated across the cell membrane, as in the commonly found cases such as high winds, droughts and drying, water migrates from its origins resulting in changes of the cell turgor pressure. Even if the water content is unchanged, or at the fresh condition, the cell turgor pressure would vary to adapt to new cellular morphologies that occur in the cases such as cell compression, tension and shear. Herein, combined with the cell turgor pressure, the cell wall and intracellular compartments govern the related cell micromechanics, which involves the study of cell’s morphological behaviour and its dynamic response. Further, based on the change of water content, a cell micromechanical study should be twofold: at the fresh state (no change of initial water content) and dehydrated/dried state.

The article "A three-dimensional (3-D) meshfree-based computational model to investigate stress-strain-time relationships of plant cells during drying" was published in 2020. Journal: PLoS One.

From a biological point of view, understanding cell micromechanics would enhance the current opinion on “*how things are happening*” inside a plant cell, enabling more detailed studies of plants. However, with the contemporary experimental procedures, investigation of cell micromechanics has been a challenging task due to diminutive spatial and temporal scales involved (typically μm length and μs time range) [2–4]. In this background, numerical modelling techniques demonstrate a promising pathway to unravel such micromechanics while encompassing the recent advancements in computational technologies, saving human effort, time and money along the way. Many numerical models have been reported in literature in this regard, which make use of various physical mechanisms and assumptions for the cellular compartments as mentioned above. Of the many numerical models developed [5–9], particle-based models have demonstrated higher ability to closely approximate the realistic nature of the cellular compartments and to elaborate their physical behaviour in a comprehensive manner.

In particle-based models, one or more cellular components (i.e. cell wall, cell fluid) are represented by a finite set of interacting particles, which carry physical properties of the respective component [10]. Loodts et.al [11] pioneered numerical modelling of plant tissues and implemented a Discrete Element Method (DEM) for the cell wall such that each discrete element corresponds to a cell wall particle. The cell fluid was not treated explicitly, apart from considering its effects through turgor pressure while allowing to evolve with cell wall dynamics. Van Liedekerke et al. [2] further improved upon this DEM model by additionally discretising cell fluid and incorporating dynamics of cell fluid along with the fluid-wall interactions. Cell fluid was modelled using Smoothed Particle Hydrodynamics (SPH), which has been a viable and popular choice to overcome remeshing issues found in classical finite element based numerical models. Through this coupled SPH-DEM meshfree-based framework, the dynamic response of a small periodic tissue under compression, tension and shear loading was predicted. Biologically, such a study is important in revealing a cell’s response with respect to changes in the environment. Further, because of the SPH computational framework, this model had the ability to simulate large deformations compared to Loodts et al. (2006) model. Later, a three-dimensional (3-D) SPH-DEM model which established the micromechanics of single fresh cell bruising was introduced [12, 13]. Micromechanics of 3-D realistic tissues that inherit a heterogeneous microstructure was also extensively studied [14]. A coupled DEM-spring mass approach was developed and a plant cell was represented as a deformable triangular mesh of fixed topology, which was subject to turgor pressure. Being computationally more efficient is one key advantage of this model, which also enabled the simulation of larger tissues. Notably, this model is limited for small deformations. This issue was addressed by Diels et al. [15], who at the same time introduced porous features of heterogenous tissues. Even at that stage, the DEM-spring mass model had limitations in providing insights to the mechanisms related to cell fluid as in SPH-DEM model.

The article "A three-dimensional (3-D) meshfree-based computational model to investigate stress-strain-time relationships of plant cells during drying" was published in 2020. Journal: PLoS One.

Generally, the SPH-DEM based models provide a detailed understanding on micromechanics compared to pure DEM based methods and coupled DEM-spring mass methods. However, the above discussed SPH-DEM based models have only been developed for fresh tissues. This raises a question: “*Can the micromechanics of dried plant cells be predicted using the results for fresh cells*?*”* or *“Does a dried plant cell behave in a significantly different manner compared to a fresh cell under mechanical stress*?”. To this end, there has been a recent development in meshfree-based plant cell drying models (see [16–21]), which proved promising capabilities over mesh-based drying models (see [22] and [23]). For example in two-dimensional (2-D) SPH-DEM drying models, a maximum of 70% moisture removal was simulated while handling non-linear large deformations of cell walls, such as wrinkling [24]. Upon the same modelling framework, 3-D drying computational models have also been reported that use the Coarse-Graining (CG) technique instead of DEM [18, 19]. The 3-D SPH-CG model has demonstrated superiority over 2-D SPH-DEM models, as it could predict up to 90% moisture removal. Additionally, such a model better represents the drying mechanisms of a cell/tissue-based three dimensional morphological description, which is more realistic [10, 19, 25]. Nonetheless, previous studies in the computational biological domain have not modelled the micromechanical behaviour of plant cells that are being dried and compressed. Consequently, the aim of this investigation has been to computationally model and simulate micromechanics of plant cells during drying using meshfree-based computational methods. In doing so, a 3-D coupled SPH-CG numerical approach has been employed to develop the model of dried plant cells that are being mechanically compressed. The micromechanical characteristics of a plant cell has been analysed in terms of stress-strain-time behaviour. The 3-D nature of the proposed model leads to a more detailed and realistic picture.

The article "A three-dimensional (3-D) meshfree-based computational model to investigate stress-strain-time relationships of plant cells during drying" was published in 2020. Journal: PLoS One.

This article has been structured as follows: Firstly, the basics of SPH-CG 3-D drying model have been discussed in Methodology, while summarising the key mathematical formulation. This section also describes the strategies to model cell compression and computational implementation. In Results and Discussion, two numerical experiments have been detailed, using apple as the model benchmark cellular material. The first experiment examines the correlations among stress, strain and time of the 3-D compressed plant cell at different levels of dryness. In each case, the predictions of the model have been assessed in comparison to experimental findings. The second numerical experiment evaluates the effects of key model parameters: initial turgor pressure, compression rate and cell wall properties on cell micromechanics. At this point, three levels of dryness are used for further elaboration of parameter sensitivity: fresh (0% dried), moderately dried (50% dried) and extremely dried (90% dried). The Conclusions section emphasizes the flexibility and potential of the proposed model for diversified computational biological investigations while highlighting limitations and potential future work.

## Methodology

### 3-D cell modelling basics

Plant biomaterials are made out of numerous different categories of cells that serve different purposes [1, 26]. These different cell categories demonstrate different behavioural characteristics even when they are subjected to the same micromechanical conditions. Nevertheless, there is the necessity for selecting a representative category of plant cells for the sake of clarity and comprehensiveness of this computational investigation. In this background, the parenchyma cells have been chosen due to the fact of being the main constituent in bulk plant ground tissues. Parenchyma cells are the living component of plant tissues while they take part in storage, photosynthesis and transport activities [27].

The article "A three-dimensional (3-D) meshfree-based computational model to investigate stress-strain-time relationships of plant cells during drying" was published in 2020. Journal: PLoS One.

Equivalent to our previously published work in this scope [18, 19], a plant cell was considered to be made out of two main components: cell fluid and cell wall. Consequently, a two-fold meshfree-based modelling approach was adopted in modelling the cell fluid and wall, mainly due to the key differences of micromechanical behaviour [19]. Cell fluid was modelled using SPH while a CG method was used for the cell wall. These two computational frameworks were numerically coupled in such a way that the pressure forces applied through the cell fluid were balanced out by the micromechanical forces created in the cell wall as per the Young-Laplace law [28, 29]. To determine the physical behaviour and interactions within and between the fluid and wall domains of a cell, a number of different force fields were adopted separately as seen in Fig 1 (a) and 1 (b). As this study uses the same basic computational configurations for a plant cell which are similar to our recently published work [19], only the novel additions to the existing micromechanical modelling framework have been presented in the main text while summarising most of the previously published information in the forthcoming tables.

**Fig 1:** The graphical summary of the coupled Smoothed Particle Hydrodynamics (SPH) and Coarse-Grained (CG) computational model proposed for simulating plant cell compression during drying. (a) Force fields in the 3-D SPH fluid model: pressure forces (***F***^***p***^), viscous forces (***F***^***v***^), wall-fluid repulsion forces (***F***^***rw***^) and wall-fluid attraction forces (***F***^***a***^); **(b)** Force fields in the Coarse-Grained (CG) 3-D wall model: stiff forces (***F***^***e***^), damping forces (***F***^***d***^), wall-fluid repulsion forces (***F***^***rf***^), wall-fluid attraction forces (***F***^***a***^), bending stiffness forces (***F***^***b***^) and wall contraction forces (***F***^***c***^); **(c)** Implementation of cell compression in the SPH-CG model through interactions between the cell wall, cell fluid and the compression plates.

### Modelling unique cell fluid mechanisms

The cell fluid was modelled as a homogeneous incompressible Newtonian fluid which demonstrates physical characteristics similar to water. However, a higher viscosity was incorporated to establish low-Reynolds-number flow characteristics while using Navier-Stokes equations to computationally model its behaviour through SPH [18, 19]. To establish the physical interactions of the cell fluid, four separate force fields were placed as shown in Fig 1(a): pressure forces (***F***^***p***^), viscous (or damping) forces (***F***^***v***^), wall-fluid repulsion forces (***F***^***rw***^) and wall-fluid attraction forces (***F***^***aw***^). It should be noted that repulsion and attraction forces have been defined in this study as Lennard-Jones (LJ) type forces. Key equations relevant to these force fields have been presented in Table 1 [19] and detailed information on each equation can be found in authors’ recent publications [19, 30]. Accordingly, in each time step, the overall force ***F***_***i***_ on a fluid particle *i* was determined as given in Eq (1). Based on this total force, the acceleration of any particle (***a***_***i***_) was then calculated using Newton’s second law of motion as given in Eq (2). Here *m*_*i*_ represents the mass of the corresponding particle. The acceleration was integrated using the leapfrog integrator [31] to determine the velocity and then the displacement.

$$F_{i}=F_{ii^{\prime }}^{p}+F_{ii^{\prime }}^{v}+F_{ik}^{rw}+F_{ik}^{aw}$$ (1)

$$a_{i}=\frac{F_{i}}{m_{i}}$$ (2)

**Table 1:** Governing equations and corresponding formulae for the fluid particle scheme [18].

Equation	Formulation	Description	References	Eq. No:
Pressure force on a fluid particle	$F_{ij}^{p}=-m_{i}\sum_{i^{\prime }}m_{j}\left(\frac{P_{i}}{\rho_{i}^{2}}+\frac{P_{i^{\prime }}}{\rho_{i^{\prime }}^{2}}\right)\nabla_{i}W_{ii^{\prime }}$	*m*: fluid particle mass *P*: cell turgor pressure *ρ*: particle density *W*: smoothing kernel *μ*: dynamic viscosity ***v***_***ii*′**_: fluid particle velocity *r*_*ii*′_: distance between particle *i* and *i*′	[12, 32]	(3)
Viscous force on a fluid particle	$F_{ij}^{v}=-m_{i}\sum_{i^{\prime }}m_{i^{\prime }}\left(\frac{\mu_{i}+\mu_{i^{\prime }}}{\rho_{i}\rho_{i^{\prime }}}\right)v_{ii^{\prime }}\frac{1}{r_{ii^{\prime }}}\frac{\partial W_{ii^{\prime }}}{\partial r_{ii^{\prime }}}$			(4)
Smoothing kernel function	$W_{ii^{\prime }}(s,h)=\frac{2}{3\pi h^{3}}\{\begin{array}{ll} \frac{2}{3}-s^{2}+\frac{s^{3}}{2} & 0<s<1\\ \frac{\left(2-s^{2}\right)}{6} & 1<s<2\\ 0 & s>2 \end{array}$	*s*: the ratio of *r*_*ii*′_/*h* *h*: smoothing length	[31]	(5)
Variable smoothing length	$h=\left(\frac{D}{D_{0}}\right)h_{0}$	*D*: current cell diameter *D*_0_: initial cell diameter *h*_0_: initial smoothing length	[33]	(6)
Equation of state (EOS)	$P_{i}\;=\;P_{T}+K[{\left(\frac{\rho_{i}}{\rho_{0}}\right)}^{7}-1]$	*P*_*T*_: initial turgor pressure *K*: fluid compression modulus *ρ*_*i*_: current density *ρ*_0_: initial density	[33]	(7)
Density–general definition	$\rho_{i}\;=\;\frac{m_{i}}{\nu_{i}}$	*m*: fluid particle mass *v*_*i*_: corresponding fluid volume	[33]	(8)
Density–time derivation	$\frac{d\rho_{i}}{dt}\;=\;m_{i}\frac{d}{dt}(\frac{1}{\nu_{i}})+\frac{1}{\nu_{i}}\frac{dm_{i}}{dt}\;=\;\frac{d\rho_{i}^{*}}{dt}+\frac{\rho_{i}}{m_{i}}\frac{dm_{i}}{dt}$	*t*: time $\rho_{i}^{*}$: density (assuming constant particle mass)	[12]	(9)
Density–SPH approximation of continuity	*$\frac{d\rho_{i}^{*}}{dt}=\sum_{i^{\prime }}m_{i^{\prime }}v_{ii^{\prime }}.\nabla_{i}W_{ii^{\prime }}=m_{i}\sum_{i^{\prime }}v_{ii^{\prime }}.\nabla_{i}W_{ii^{\prime }}$*		[31, 33]	(10)
Rate of mass transfer	$\frac{\;dm_{i}}{dt}\;=\;-\frac{A_{c}L_{p}\rho_{i}}{n_{f}}(P_{i}+\;\Pi )\;$	*A*_*C*_: *cell wall surface area* *L*_*P*_: cell wall permeability *Π*: *osmotic potential* *n*_*f*_: *number of fluid particles*	[1]	(11)
Wall-fluid repulsion force (LJ)	*$F_{ik}^{rw}=\sum_{k}f_{ik}^{rw}x_{ik}$*	$f_{ik}^{rw}$: *magnitude of the force* ***x***_***ik***_: *position vector*	[12, 16, 31]	(12)
Wall-fluid attraction force (LJ)	*$F_{ik}^{aw}=\sum_{k}f_{ik}^{aw}x_{ik}$*	$f_{ik}^{aw}$: *magnitude of the force* ***x***_***ik***_: *position vector*		(13)

The article "A three-dimensional (3-D) meshfree-based computational model to investigate stress-strain-time relationships of plant cells during drying" was published in 2020. Journal: PLoS One.

### Modelling unique cell wall mechanisms

Cell walls gain their structural integrity through biopolymeric constituents like cellulose, hemicellulose and pectin [34–36]. Consequently, their micromechanical behaviour could not be modelled with simple linear stress-strain-time relationships [37]. In this study, a CG method have been used to computationally model the cell wall segment of the plant cells [19]. To incorporate the physical interactions of the cell wall model, six separate force fields were applied: stiff forces (derived from harmonic potential) (***F***^***e***^), damping forces (***F***^***d***^), wall-fluid particle repulsion forces (***F***^***rf***^), wall-fluid particle attraction forces (***F***^***af***^), bending stiffness forces (***F***^***b***^) and wall contraction forces (***F***^***c***^) [16, 19, 33]. Accordingly, the total force (***F***_***k***_) on a wall particle *k* was be determined as in Eq (14). As described in the previous section for fluid particles, Newton’s second law of motion was then employed to determine the acceleration of each wall particle based on ***F***_***k***_. A summary of the key equations have been presented in Table 2 [19] and detailed information on each equation can be found in authors’ recent publications [19, 30].

$$F_{k}=F_{kj}^{e}+F_{kj}^{d}+F_{ki}^{rf}+F_{ki}^{af}+F_{kj}^{b}+F_{kj}^{c}$$ (14)

**Table 2:** Governing equations and corresponding formulae for the wall particle scheme.

Equation	Formulation	Description	References	No:
Stiff force on a wall particle	$F_{kj}^{e}\;=\;\frac{Gl_{0}t_{0}}{\sqrt{3}}(\lambda -\frac{1}{\lambda^{5}})n$	G: shear modulus (≈ *E*/3) *E*: Young’s modulus *λ* = *l*/*l*_0_: current stretch ratio *l*: current length *l*_0_: initial length *t*_0_: cell wall thickness ***n***: unit normal vector	[8]	(15)
Damping force on a wall particle	$F_{kj}^{d}\;=\;-\gamma \nu_{kj}$	*γ*: damping constant ***v***_***kj***_: relative velocity	[16]	(16)
Wall-fluid repulsion force (LJ)	$F_{ki}^{rf}\;=\;f_{ki}^{rf}x_{ki}$	$f_{ki}^{rf}$: magnitude of the force ***x***_***ki***_: position vector	[12, 16, 31]	(17)
Magnitude of wall fluid repulsion force	*$f_{ki}^{rf}=\{\begin{array}{ll} f_{0}^{rf}\left[{\left(\frac{r_{0}}{r_{ki}}\right)}^{8}-{\left(\frac{r_{0}}{r_{ki}}\right)}^{4}\right]\left(\frac{1}{r_{ki}{}^{2}}\right) & \left(\frac{r_{0}}{r_{ki}}\right)\geq 1\\ 0 & \left(\frac{r_{0}}{r_{ki}}\right)<1 \end{array}$*	*r*_0_: initial gap *r*_*ki*_: current gap $f_{0}^{rf}$: LJ contact strength	[12, 16, 31]	(18)
Wall-fluid attraction force (LJ)	$F_{ik}^{af}=\sum_{k}f_{ik}^{af}x_{\text{ik}}$	$f_{ik}^{af}$: magnitude of the *force* *x*_*ik*_: position vector	[12, 16, 31]	(19)
Bending force on wall particles	**$F^{b}=-\frac{k_{b}}{2}\frac{\partial }{\partial x}\sum_{i=1}^{N}L_{n}\frac{1-{\hat{n}}_{ijk}\cdot {\hat{n}}_{ilj}}{1+{\hat{n}}_{ijk}\cdot {\hat{n}}_{ilj}}$**	*k*_*b*_: bending stiffness ${\hat{n}}_{ijk}$ and ${\hat{n}}_{ilj}$: unit normal vectors *L*_*n*_: a geometry specific parameter *x*: distance	[19]	(20)
Wall contraction force	$F_{kj}^{c}\;=\;k_{wc}[L-L_{0}^{\prime }[1-\frac{a}{b}(1-\frac{X}{X_{0}})]]$	*k*_*wc*_: force coefficient for wall contractions *L*: current width of a wall element $L_{0}^{\prime }$: width of the wall element at the fully turgid condition *a*,*b*: empirical parameters *X*/*X*_0_: normalised moisture content	[19]	(21)

The article "A three-dimensional (3-D) meshfree-based computational model to investigate stress-strain-time relationships of plant cells during drying" was published in 2020. Journal: PLoS One.

### Modelling cell compression

Cell compression was modelled as a simulation of restricting the cell (both fresh and dried) between two flat plates based on comparable experimental and numerical investigations reported in the literature [8, 38]. The comparable experimental investigation was a compression test conducted on an *in vitro* plant cell to analyse the corresponding mechanical properties. The comparable numerical investigation was a particle-based model that simulated micromechanics of single fresh cells, which was validated through the findings of the aforementioned experimental investigation. Thus in this article, a similar method has been incorporated to the meshfree-based SPH-CG computational framework to model the micromechanical response of dried plant cells [18, 19].

The compression was implemented by placing two horizontal plates, one at the bottom of the cell and the other at the top as seen in Fig 1(c). The bottom plate remained static at its position while the top plate was moved downwards gradually. The physical interactions between the cell wall and compression plates were established through a force-field: plate-wall force (***F***^***pw***^). When the CG particles in the wall overlaps with the critical distance region of the compression plates (*r*^*pw*^), each overlapping wall particle is repelled by a force. The magnitude of this force is proportional to the difference between *r*^*pw*^ and the current distance between the wall particle and the plate (see Fig 1(c)). It should be noted that ***F***^***pw***^ has been defined as a vertical force due to the orientation of the compression mechanism. The force on a wall particle (***F***^***pw***^) due to compression has been calculated as,

$$F^{pw}=\;-k_{pw}\Delta x_{pw}$$ (22)

where *k*_*pw*_ is the force coefficient for the force-field and Δ***x***_*pw*_, the difference between *r*^*pw*^ and the current distance between the wall particle and the plate. The negative signifies that force on the wall exerted by the compression plate is in the opposite direction to the positive vertical direction. The velocity of the moving compression plate (top) was set at a sufficiently low rate in order to minimise any inertial effects imposed on the cell which might lead to unrealistic and unstable results in terms of morphological and micromechanical response.

The article "A three-dimensional (3-D) meshfree-based computational model to investigate stress-strain-time relationships of plant cells during drying" was published in 2020. Journal: PLoS One.

With the addition of the plate-wall force, ***F***^***pw***^, the total force on a wall particle, ***F***_***k***_, can be given as in Eq (23) below.

$$F_{k}=F_{kj}^{e}+F_{kj}^{d}+F_{ki}^{rf}+F_{ki}^{af}+F_{kj}^{b}+F_{kj}^{c}+F_{k}^{pw}$$ (23)

where $F_{k}^{pw}$ is the force on a wall particle exerted by the compression plates. Since the effect of pressure is relative, a gauge pressure value was used for the turgor pressure while assuming the atmospheric or outside pressure to be zero. This way, the used turgor pressure value becomes the actual pressure difference across the cell wall. Further, the plate-wall force (***F***^***pw***^) contributes as the external boundary condition to the cell wall acting in the vertical direction on the interacting wall-plate particle-pairs. This force is defined as a repulsion force that is directly proportional to the difference between *r*^*pw*^ and the current distance between the wall particle and the plate (see Fig 1(c)). In addition, the interactions between cell wall and fluid particles have been defined through Lennard-Jones (LJ) type forces: wall-fluid repulsion forces (***F***^***rw***^ and ***F***^***rf***^) and wall-fluid attraction forces (***F***^***aw***^ and ***F***^***af***^) [8, 12].

The article "A three-dimensional (3-D) meshfree-based computational model to investigate stress-strain-time relationships of plant cells during drying" was published in 2020. Journal: PLoS One.

### Modelling cellular deformation under different turgor pressures

Water plays a critical role in the life of plants and plant cells, similar to any other living organism [1]. Turgor pressure is the fluid pressure built inside plant cells due to the inherent water-balancing functionality of the semi-permeable cell wall membrane. It is crucial for many physiological processes of plants such as cell growth, gas exchange and transport. In addition, turgor pressure is vital for the rigidity and mechanical stability of plant tissues. Subsequently, it is an essential parameter in determining their morphological behaviour. This was taken into consideration in our recent computational modelling studies that looked into plant cells’ morphological behaviour during drying [18, 19]. However, those studies have not yet evaluated the effects of significant turgor pressure changes in plant cells towards the morphological response. In this study, this phenomenon has been addressed in a detailed manner. In addition, the effects of significant turgor pressure variations on the stress-strain relationship of cells have been investigated comprehensively. In doing so, cells with different turgor pressures were computationally modelled and their morphological response as well as the stress-strain relationships were observed simultaneously. The experimentally determined standard turgor pressure of apple cells (i.e. 200 kPa) was taken as the benchmark in this turgor pressure sensitivity analysis. Concurrently, a turgor pressure of 100 kPa was considered as the low turgor pressure while 300 kPa was the high turgor pressure.

### Numerical implementation of the cell model

The numerical implementation of this meshfree-based cell micromechanics model consisted of two main stages: the drying stage and the compression stage. The drying stage was computationally implemented similar to our previously published work [18, 19]. The compression stage was implemented using the mathematical formulation discussed in the previous section. The cell was initialised with a particle scheme consisting of 3082 fluid particles (SPH) and 2067 wall particles (CG). Further details on the suitability of these particle numbers have been evaluated in detail in our recent publication [18]. The model equations relating to the drying and compression processes were embedded with necessary physical, biological and geometrical parameters for a parenchyma cell of a Royal Gala apple (*Malus Domestica*) as given in Table 3. This particular type of apple cells was specifically selected due to the availability of experimental findings on stress-strain relationships for model validation purposes.

The article "A three-dimensional (3-D) meshfree-based computational model to investigate stress-strain-time relationships of plant cells during drying" was published in 2020. Journal: PLoS One.

**Table 3:** Physical, biological and geometrical property values used for the 3-D single cell compression model, representing an apple cell (Royal Gala apple (*Malus Domestica*)).

Parameter	Value	Reference
Initial cell radius [μm]	75	[39]
Cell wall shear modulus (*G*) [MPa]	18	[40]
Initial thickness of the cell wall (*t*) [μm]	6	[40]
Initial cell fluid mass [kg]	1.767 × 10^−9^	Set ([16])
Initial cell wall mass [kg]	1.767 × 10^−10^	Set ([16])
Cell wall damping ratio (*γ*) [Ns/m]	5 × 10^−6^	Set ([16])
Cell fluid viscosity (*μ*) [Pas]	0.1	Set ([12, 13])
Initial SPH smoothing length (*h*_*0*_) [μm]	6.8	Set ([12, 16, 31])
Turgor pressure of fresh cell (*P*_*T*_) [kPa]	200	[38]
Osmotic potential of fresh cell (*-π*) [kPa]	- 200	Equal to—P_T_ ([12, 16])
Cell wall permeability during drying (*L*_*P*_) [m^2^s/N]	2.5 × 10^−6^	Set [1]
Cell wall permeability during compression (*L*_*P*_*’*) [m^2^s/N]	1.0 × 10^−12^	[1]
Cell fluid compression modulus(*K*) [MPa]	20	Set ([16])
Number of fluid particles (*N*_*f*_)	3082	Set
Number of wall particles (*N*_*w*_)	2067	Set
LJ contact strength for attraction forces ${\;(f}_{0}^{a})$ (Nm^-1^)	1 × 10^−11^	Set
LJ contact strength for repulsion forces ${\;(f}_{0}^{r})$ (Nm^-1^)	5 × 10^−12^	Set
Cell wall bending stiffness (*k*_*b*_) [Nmrad^-1^]	1.0 × 10^−10^	Set ([24])
Cell wall contraction force coefficient (*k*_*w*c_) [Nm^-1^]	1.0 × 10^4^	Set ([24])
Plate-wall force coefficient (*k*_*pw*_*)* [Nm^-1^]	1.0 × 10^3^	Set
Plate length *x* width [μm]	150 × 150	Set
Time step for numerical implementation (Δ*t*) (ns)	1	Set
Number of time steps for drying	50000	Set
Number of time steps for compression	25000	Set

A leapfrog integrator [31, 41] was used for the numerical integration with a time-step optimised using the Courant-Friedrichs-Lewy (CFL) stability criterion [8, 42, 43]. The cell was allowed to inflate (fresh condition) or deflate (dried conditions) depending on the dryness level. Once the cell reached its steady state in the corresponding dryness level, the compression of the cell was initiated using two flat plates as previously described. During the drying phase, a higher than usual magnitude was used for the cell wall permeability (*L*_*P*_) to improve the computational efficiency of the model (*L*_*P*_ = 2.5 × 10^−6^). This was a method followed by previous researchers [16] without any undesirable consequences on the actual results of the model. With the commencement of compression stage, the magnitude of this parameter was changed to its real value (*L*_*P*_*’* = 1.0 × 10^−12^). Based on this *L*_*P*_ variation, there is a significant change of mass transfer rate across the cell wall for the drying and compression stages as governed by Eq (11). The effects of this mass transfer rate variation have been discussed in the upcoming sections of this article.

The article "A three-dimensional (3-D) meshfree-based computational model to investigate stress-strain-time relationships of plant cells during drying" was published in 2020. Journal: PLoS One.

The force-displacement information of the cell was recorded continuously. And this data was then used to establish corresponding stress-strain-time relationships. The results were compared to equivalent findings from relevant experimental investigations. The source code for the computational model was coded in C++ programming language and executed in the High-Performance Computing (HPC) facility at the Queensland University of Technology (QUT), Brisbane, Australia. Open Visualisation Tool (OVITO) [44] was used for the visualisation of post-processed computational data.

## Results and discussion

### Numerical experiments 1: Basic micromechanics

#### Computational modelling of drying of a single 3-D cell

In order to observe the geometrical shrinkage and other micromechanics during drying, initial simulations on gradual drying of an apple cell was carried out and the subsequent results are shown in Fig 2(a). During drying, in response to the gradual reduction of turgor pressure, the cell deflates to a certain extent. This cell geometrical deflation or shrinkage can be clearly observed by comparing the gap between the black coloured line (plate) and the cell wall in Fig 2(a), where the gap has gradually increased as the degree of dryness increases (i.e. *X/X*_*0*_ decreases). However, cell wall wrinkling cannot be observed since the cell is relatively free from other external influences and there is a positive turgor pressure value still keeping the cell wall in tension, which is in alignment with authors’ recently published work [16].

**Fig 2:** SPH-CG model predictions for (a) uncompressed and (b) compressed dried cells at different dryness levels at normal turgor pressure (200 kPa). (*X/X*_*0*_ is the normalised moisture content).

#### Computational modelling of compression of a single 3-D cell

In Fig 3, the morphological behaviour of the cell model with simulation time has been demonstrated. When the fresh cell is being compressed between two parallel plates, it is evident that the cell deforms in a stiff manner, shifting from the an almost pure-spherical shape into a top-and-bottom-flat shape causing higher stresses and strains in the cell wall. Turgor pressure and external deformations can be given as the key reasons for the increased stresses and strains. Compared to the fresh cell, the dried cells (*X/X*_*0*_ = 0.5 and 0.1) indicate lower stiffness characteristics with lower strain and stress occurrences during the deformation process. This is an indication that the forces required to deform a dried cell will be smaller compared to a fresh and more turgid cell, particularly if the cell undergoes a finite amount of deformation from its original shape. This behaviour is naturally expected in a typical dried food processing operation, commonly observed in the food industry where cellular damage will not be readily entertained. Here, the maximum strain amount was limited compared to the original vertical diameter of the fresh cell. However, based on the merits of the meshfree nature of this 3-D computational cell model, extreme deformations of cells can be simulated, even rupturing the cell wall in extreme loading conditions [8]. Although such scope was not intended in this study, the authors propose that it is quite possibly a target for prospective further research.

The article "A three-dimensional (3-D) meshfree-based computational model to investigate stress-strain-time relationships of plant cells during drying" was published in 2020. Journal: PLoS One.

**Fig 3:** Depiction of gradual compression of dried cells as predicted by the 3-D SPH-CG model. (a) fresh cells (*X/X*_*0*_ = 1.0); (b) dried cells (*X/X*_*0*_ = 0.5); (c) dried cells (*X/X*_*0*_ = 0.1) (*X/X*_*0*_ is the normalised moisture content.

Fig 2(b) visualises the model predictions for a compressed cell corresponding to all the dryness levels. It demonstrates that when the degree of dryness increases, there is less resistance to compression. The flat area of the cell wall which interacts with the plate becomes smaller as the cell gets dried. The main driving force for this behaviour can be argued as the lower turgor pressure of the cell fluid causing less resistance towards compression force exerted by the compression plate. This trend can be clearly witnessed by comparing the fresh condition and the extremely dried condition of Fig 2(b), where the horizontal axis size of the cell has reduced in a qualitatively observable manner, implying the dried cell’s less strained deformations due to its default contracted geometry. Further, relatively higher wrinkling taking place closer to the plates, such as the roundness of the corner formed in the cell wall near the plates, which become relatively less rounded in the case of extreme dryness levels (e.g. *X/X*_*0*_ ≤ 0.3). Specific areas of the simulations have been magnified and visualised in Fig 2(b) to elaborate this behaviour. Upcoming sections will present more quantitative comparisons of stresses and strains of cell walls in plate compression, drawing more specific insights towards the corresponding micromechanical behaviour.

To further quantify the morphological variation of the cell model when going through drying and compression, the cell surface area and volume were analysed. Fig 4(a) gives the cell surface area variation during drying and compression. During the simulations, cell area was calculated by summing up all the areas enclosed by the cell wall particle network. Accordingly, for all the dryness levels presented here (*X/X*_*0*_ = 1.0, 0.5 and 0.1), there is a significant variation of the cell surface area at the very beginning of the simulation (0–4 μs). This variation can be attributed to the significantly high moisture transfer that occurs across the cell wall due to the difference between the osmotic potential and the dynamically varying turgor pressure compared to the respective initial states. After this initial settling of the models, a relatively stagnant phase can be observed in both drying and compression stages. Towards the end of the compression stage (70–75 μs), there is a slight increase of surface area. This increment is more dominant in the fresh condition compared to the dried states. The major reason behind this variation is the change of shape of the cell due to compression. In other words, the cell transforms from an almost pure-spherical shape into a top-and-bottom-flat spherical shape (see Fig 3) as discussed above. This top-and-bottom-flat nature becomes further intensified with increasing compression giving rise to a further rise of surface area. The change of cell wall permeability (*L*_*P*_) during the compression period and subsequent changes in the mass transfer rate (previously explained in the *Numerical implementation of the cell model* sub-section) could also be given as a contributing factor to this area variation observed towards the end of compression stage.

The article "A three-dimensional (3-D) meshfree-based computational model to investigate stress-strain-time relationships of plant cells during drying" was published in 2020. Journal: PLoS One.

**Fig 4:** The variation of (a) cell surface area; and (b) cell volume during drying and compression for different dryness levels at a typical turgor pressure of 200 kPa. (*X/X*_*0*_ is the normalised moisture content).

The volume variation of the cell during drying and compression is given in Fig 4(b). A rise of volume can be observed at the beginning of the drying stage (0–4 μs). The volume increment is more pronounced at higher moisture levels (e.g. *X/X*_*0*_ = 1.0). This rise of volume occurs due to the dynamic balance between turgor pressure and cell wall hoop stress as per Young-Laplace law [28, 29]. The rate of moisture transport across the cell wall affects this phenomenon as well [12]. The initial rise of volume is followed by a steadier phase until the end of drying period through to the compression stage for all the dryness levels which is an equivalent behaviour to the above discussed cell surface area variation. Towards the end of the compression stage (70–75 μs), a slight decrease in cell volume can be observed. This slight reduction can be mainly attributed to the changed cell shape and the magnitude of *L*_*P*_ as previously discussed. Based on these insights provided by Fig 4, it can be concluded that cell surface area and volume are not conserved at either of the drying or compression phases.

The article "A three-dimensional (3-D) meshfree-based computational model to investigate stress-strain-time relationships of plant cells during drying" was published in 2020. Journal: PLoS One.

It should be noted here that the cell has been thermodynamically considered as an open system with a semi-permeable boundary (i.e. cell wall) similar to the previously published work [16, 19]. Consequently, mass and energy cross the cell wall at different stages of the simulation (e.g. drying and compression). During the time evolution of the cell model, moisture crosses the cell wall from cell fluid to the external environment leading to turgor pressure variations until cell reaches steady state with no more mass transfer nor turgor pressure variation [8, 12, 19]. Mass transfer from the cell was represented as reductions of mass of fluid particles, without any physical escape of particles across the cell wall. This means that cell mass is not conserved during the drying and compression stages, which is similar to the actual plant cells [19, 33]. Cell wall permeability (*L*_*P*_) is a critical parameter that influences the overall mass transfer at any stage of drying or compression [18].

### The variation of stress and strain with time

To demonstrate the variation of stress and strain with the gradual deformation of the cell under compression, the strain variation of the cell with time has been plotted in Fig 5. As the cell is gradually compressed, the average strain variation of the cell demonstrates a two-step behaviour: initial non-linear stage, followed by a linear stage for a longer time period during the final stages of the compression. Interestingly, this behaviour can be commonly observed in all the dryness levels (i.e. different *X/X*_*0*_ levels). It implies that the cell fluid tends to reach a sufficiently higher turgor pressure value after a certain level of compression, causing the cell wall to be in tension. This causes the cell to respond in a stiffer manner. In the initial phase, the behaviour of the cell is such that the strain gradually increases leading to steady local peaks. The cells with higher turgor pressures lead to higher strains. Still, the peak strain values initially drop for short time intervals even though they eventually increase at later stages due to compression. The cells with higher turgor pressures tend to lose the strain more quickly, while dried cells tend to have a slow strain release and reach a relatively lower strain level compared to the turgid cells. However, it should be noted that the fresh cells exhibit a minimum strain in the order of 0.035, which is still higher than that of the dried cells, ranging from 0.005 to 0.025. The strain variation rate is approximately similar for all the dryness levels as seen from gradients in the curves of Fig 5.

The article "A three-dimensional (3-D) meshfree-based computational model to investigate stress-strain-time relationships of plant cells during drying" was published in 2020. Journal: PLoS One.

**Fig 5:** Variation of average strain with time during compression simulation of the SPH-CG cell drying model at a turgor pressure of 200 kPa. (*X/X*_*0*_ is the normalised moisture content).

The inertial effects of the top plate making initial contact with the cell during the compression process could be given as a key reason behind the initial non-linear stage of strain variation of the cell observed around the 52–62 μs period (see Fig 5). To further elucidate this aspect, it would be helpful to understand the process of cell compression which was undertaken in this study in more detail. At the beginning of the cell compression simulation, the top plate was placed above the cell with a certain gap so that this initial setup could be used with cells of multiple sizes. In other words, the top plate was not contacting the cell at the beginning of compression simulation. With time, the top plate was moved gradually through this gap towards the cell at a certain velocity as described previously in the *Modelling cell compression* sub-section. When the top plate makes the initial contact with the top part of the cell, there is a certain lag phase of force transmitting to the cell through acceleration of particles which were static prior to the contact (pre-contact). Similar behaviours have been observed previously by other researchers who have been working on computational modelling investigations of cells [8]. It is during this lag phase when the initial non-linear phase strain variation occurs. Following this lag phase (post-contact), the cell deforms gradually in synchronisation with the plate which corresponds to the linear strain variation seen in Fig 5. This has been visualised using cell and plate locations at different stages of compression in Fig 5. Based on the mechanics involved with this phenomenon, there could also be effects of cell wall damping ratio (*γ*) and fluid viscosity (*μ*) towards such dynamics where little research has been conducted so far. Even though such an investigation could be well implemented using the proposed SPH-CG computational approach, such additional work remains out of the scope of this paper while leading to relevant future work.

The cell stress variation with time is shown in Fig 6. During compression, the stress variation of the dried cell demonstrates a non-linearly increasing behaviour for the entire period of simulation with local peaks, which is a common trend for all the dryness levels. This implies that the rate of stress-rise increases with time. However, the rate of stress-rise is not the same for all dryness levels, where it is higher for lower dryness levels (i.e. high *X/X*_*0*_ levels) and it is lower for higher dryness levels. Even though a more linear behaviour was observed for cell wall strain as per Fig 6, the non-uniform increase of the stress observed from Fig 6 could be a result of the non-linear stress-strain relationship used in developing the CG cell wall model. This relationship has been detailed in Eq (15) in Table 2. The local peaks correspond to the initial non-linear strain variation stage discussed in the strain-variation section above with respect to Fig 5. There is a certain lag phase defined by force transmission and inertial effects to be observed in the stress variation (see Fig 6) during the same time period (52–62 μs period approximately).

The article "A three-dimensional (3-D) meshfree-based computational model to investigate stress-strain-time relationships of plant cells during drying" was published in 2020. Journal: PLoS One.

**Fig 6:** Variation of stress with time during the compression simulation of the SPH-CG cell drying model at a turgor pressure of 200 kPa. (*X/X*_*0*_ is the normalised moisture content).

### Stress-strain relationships for cells under compression

The stress-strain relationship simulated by the SPH-CG computational model for an apple cell going through drying and compression is given in Fig 7. Relevant experimental results have also been considered for the validation of model predictions. The gradient of each stress-strain curve is an approximate indication of the magnitude of cell stiffness. It can be seen that the increasing level of dryness (i.e. decreasing normalised moisture content (*X/X*_*0*_) values) leads to gradual reductions of the overall compressive stiffness. For example, the fresh cell (i.e. *X/X*_*0*_ = 1.0) demonstrates a higher compressive stiffness (i.e. gradient of the curve). This characteristic could be equivalently observed in the experimental findings as well, where the experimental curve for the fresh apple cells (from the study of Oey et al. [45]) demonstrates a relatively higher stiffness relative to the experimental curve for dried cells (from the study of Lewicki et al. [46]). It further indicates that higher resistive forces should be expected when processing fresh and turgid food plant materials compared to processing comparable dried versions. Accordingly, the turgor pressure can be identified as a key factor governing the force fields involved in processing food plant materials.

**Fig 7:** Comparison of model predictions for stress-strain relationship of the plant cell (at normal turgor pressure: 200 kPa) with corresponding experimental findings. [45, 46].

It could also be observed that at the extreme levels of dryness (e.g. *X/X*_*0*_ = 0.1 and 0.3), there is a higher level of cell wall stiffness demonstrated by the cell at the latter part of compression (strain > 0.1). In other words, the compressive stiffness of the cell with a *X/X*_*0*_ value of 0.1 is higher compared to that of the cell with a *X/X*_*0*_ value of 0.3. This is clearly not the case for relatively less-dried cell simulations (e.g. *X/X*_*0*_ *=* 0.9, 0.7 and 0.5). To make this clearer, the markers from all the curves have been removed in Fig 7. This indicates the stress-strain curve corresponding to *X/X*_*0*_ value of 0.1 staying above the curve corresponding to the adjacent higher moisture content (i.e. *X/X*_*0*_ = 0.3). The reason behind this could be the default shrinkage or hardening of the cell wall solid structure coming into effect as the cell becomes extremely dried [9]. This has been incorporated as the cell wall contraction forces of the cell wall model (see Eqs (14) and (21)), which is intensified in the case of extremely dried conditions. At higher moisture contents, the solid structure of the cell wall might not be affected significantly due to the abundant availability of free moisture in the cell. However, at the extreme dryness levels, the lack of free moisture could be leading to significant alterations of the cell wall solid structure as demonstrated by the meshfree-based computational, biological and micromechanical framework used in this study.

The article "A three-dimensional (3-D) meshfree-based computational model to investigate stress-strain-time relationships of plant cells during drying" was published in 2020. Journal: PLoS One.

As seen in Fig 7, there is a certain discrepancy between the model predictions and experimental findings, specifically at high strain values. The key reason behind this general discrepancy can be identified as the lack of cell-cell interactions and intercellular spaces in the current proposed computational modelling approach. In reality, the effects from neighbouring cells and intercellular spaces have a crucial role to play in the micromechanical as well as morphological behaviour of one single cell. These intercellular effects are embedded in the experimental findings employed in this investigation. This highlights the importance of further extending this computational approach into multicellular and large tissue scales. The resulting models will have an enhanced potential to better replicate the true stress-strain behaviour of plant cellular materials.

### Numerical experiments 2: Sensitivity analyses

#### Sensitivity of cell behaviour towards turgor pressure

Fig 8 shows the 3-D SPH-CG model predictions for compression of dried cells at different turgor pressures. As per experimental sources in literature, the typical turgor pressure of a fresh (or turgid) apple cell is approximately 200 kPa [40]. Based on that premise, to simulate a high-turgor pressure condition of a cell, 300 kPa pressure was used which is 150% of the average turgor pressure. Similarly, for a low turgor pressure simulation, a 100 kPa pressure was used which is 50% of the average turgor pressure. By comparing Fig 8(a), 8(b) and 8(c), there is little difference between fresh conditions. However, a slightly larger cell geometry can be observed in the case of the extremely dried condition (*X/X*_*0*_ = 0.1). Also, as the cell turgor pressure increases, the curvature of the edge formed on the cell wall next to the plate-touching region tend to become higher.

The article "A three-dimensional (3-D) meshfree-based computational model to investigate stress-strain-time relationships of plant cells during drying" was published in 2020. Journal: PLoS One.

**Fig 8:** SPH-CG model predictions for compression of dried cells at different dryness levels. at: (a) high turgor pressure (300 kPa); (b) normal turgor pressure (200 kPa); (c) low turgor pressure (100 kPa). The blue dashed lines have been placed in order to facilitate the efficient identification of morphological changes among different turgor pressures. (*X/X*_*0*_ is the normalised moisture content).

The graphs of stress-strain relationships at different turgor pressures and different dryness levels have been presented in Fig 9. In these graphs, the SPH-CG model predictions as well as comparable experimental findings [45, 46] for cell compression scenarios have been presented. Fig 9(a) shows results for high turgor pressure while Fig 9(b) and 9(c) correspond to typical and low turgor pressure, respectively. As seen in Fig 8, there are no significant variations of cell morphological changes among different turgor pressures. It should be noted that there are no comparable changes in cell diameter, area or cell wall wrinkling as demonstrated by different visualisations in Fig 8. This characteristic is observed to be true for all the dryness levels (i.e. 0.1 ≤ *X/X*_*0*_ ≤ 1.0). Nevertheless, there seems to be significant quantitative variations in cell stress-strain behaviour at different turgor pressures as seen in Fig 9.

**Fig 9:** The stress-strain relationships demonstrated by the SPH-CG cell computational model at different dryness levels. at: (a) high turgor pressure (300 kPa); (b) normal turgor pressure (200 kPa); (c) low turgor pressure (100 kPa). (*X/X*_*0*_ is the normalised moisture content).

As discussed previously, the trend of stiffness reduction with increasing dryness levels is present at all three turgor pressures studied in this investigation. The absolute stiffness of fresh cells going through compression predicted by the developed SPH-CG model seems to be increasing with increasing turgor pressure. This means that for the lower turgor pressure, the stiffness demonstrated during cell compression is lower particularly at the low dryness levels. However, with the increasing dryness level, the stiffness variation among cell-models of different turgor pressures is observed to be declining (see Fig 9(a) and 9(c)).

The article "A three-dimensional (3-D) meshfree-based computational model to investigate stress-strain-time relationships of plant cells during drying" was published in 2020. Journal: PLoS One.

To investigate this phenomenon further, the graphs in Fig 10 were created by plotting the stress-strain relationships for all three turgor pressures (i.e. Normal: 200 kPa, High: 300 kPa, Low: 100 kPa) in one graph particularly for the fresh cell state (*X/X*_*0*_ = 1.0) and extremely dried cell state (*X/X*_*0*_ = 0.1). Fig 10 confirms the stiffness rise with increasing turgor pressure at the fresh cell state. For example, the stiffness of the fresh cell at 300 kPa seems to be significantly higher compared its 100 kPa counterpart. However, the stiffness variation at the extremely dried state seems to be negligibly smaller. All three stress-strain curves at *X/X*_*0*_ = 0.1 for different turgor pressures are virtually overlapping.

**Fig 10:** The stress-strain relationship of fresh (*X/X*_*0*_ = 1.0) and extremely dried (*X/X*_*0*_ = 0.1) cells at different turgor pressures. (i.e. Normal: 200 kPa, High: 300 kPa, Low: 100 kPa) (*X/X*_*0*_ is the normalised moisture content).

With decreasing turgor pressure, the fresh cell stress-strain curves are approaching its experimental counterpart as seen in Fig 10. In other words, the stiffness of the cell at 100 kPa seems to be closer to the stiffness of the experimental findings for the fresh cell. However, this characteristic is not predominant at the extremely dried state of the cell. The implication of this seems to be that apart from the turgor pressure, there are other properties of the developed SPH-CG computational model that contribute towards the closer approximation of true micromechanical behaviour of cells.

It should also be noted that for the dryness levels considered, there is a significant difference between the SPH-CG model predictions and the corresponding experimental findings as seen from Figs 9 and 10. This can be explained through two main reasons. Firstly, whether they are fresh or dried, cells are not present as single and separate units in real plant tissues. Instead, they are bonded in large numbers through middle lamella [1]. At its current formulation, since the proposed is a single cell model, for any dryness level, the cell-cell interactions have not yet been taken into consideration. Experimental results obviously represent behaviours of plant tissues, not single cells. This difference is one major reason behind the discrepancy between model predictions and experimental findings as seen in Figs 9 and 10 [18]. The movement and shrinkage of cells in real plant tissues are restricted as each cell is bonded in almost all directions to the surrounding cells through a pectin layer [1]. This suggests that the gradient of a tissue model stress-strain curve would be significantly less for all dryness levels compared to model predictions for a single cell as seen in Figs 9 and 10. In other words, the agreement between the model predictions and experimental findings can significantly improve for a tissue model. Furthermore, bulk scale properties such as case-hardening and heterogeneity certainly come into play during experiments [7]. The absence of such properties could play a role in this difference between the model predictions and experimental results. The proposed SPH-CG single cell model has proven potential to be extended to tissue scale [18] which can provide the opportunity to incorporate the cell-cell interactions and bulk scale properties while leading to further future work.

The article "A three-dimensional (3-D) meshfree-based computational model to investigate stress-strain-time relationships of plant cells during drying" was published in 2020. Journal: PLoS One.

Secondly, this discrepancy between model predictions and experimental findings could be attributed to the absence of plasticity in the cell wall model. In the proposed model, cell wall has been considered to behave in an elastic manner. Previously published work in this domain has shown that combining plastic deformation characteristics with the existing elastic behaviour could improve the agreement of the model predictions with experimental findings [13, 47]. In other words, a hybrid elastic-plastic mechanical behaviour has potential to better approximate the experimental findings. Combining such an enhanced wall model into the proposed 3-D SPH-CG computational cellular framework was not considered in this study as the main focus here was to investigate drying related morphological changes of plant cells rather than evaluating finer characteristics of plant cell walls and related mechanisms.

#### Sensitivity of cell behaviour towards strain rate

Fig 11 demonstrates the stress-strain relationship of the cell at different compression rates at different levels of dryness. With increasing compression rates, there are local peaks of stress, even at low levels of strain. The higher the compression rate, the more prominent the impulsive increment of stress during the compression process. This behaviour can be observed in a pronounced manner at a top plate velocity of 10.0 ms^-1^ compared to lower velocities. These sudden peaks of stress could be arising due to the more impulsive nature of force application generated through higher compression rates (plate velocities). This demonstrates the effects of inertial impacts due to the application of compressive force through the compression plate, which is further evident through the significant reduction of stress after initial peaks.

**Fig 11:** The stress-strain relationship of cells as affected by varying compression rates. (a) fresh cells (*X/X*_*0*_ = 1.0); (b) moderately dried cells (*X/X*_*0*_ = 0.5); (c) extremely dried cells (*X/X*_*0*_ = 0.1) (*X/X*_*0*_ is the normalised moisture content).

The article "A three-dimensional (3-D) meshfree-based computational model to investigate stress-strain-time relationships of plant cells during drying" was published in 2020. Journal: PLoS One.

Fig 12 shows the variation of stress with time during cell compression simulation as affected by varying compression rates, which further validates the conclusions made through Fig 11. That is, with increasing compression rate, the inertial effects play a more critical role in the stress-strain behaviour demonstrated by the cell. However, as seen in Fig 11(b) and 11(c) as well as Fig 12(b) and 12(c), the intensity of the impulsive nature reduces with increasing dryness levels. Nevertheless, the relative nature of the inertial effects still exists at varying compression rates. This is a novel insight derived through this study which could be taken into consideration when designing and implementing industrial drying processes for fruits, vegetables or any other plant biological material. For example, due to the increased inertial effects and the subsequent impulsive nature of the force application, the food cellular structure could be damaged. This could clearly affect the quality of the dried food product in terms of texture and visual appeal as well as nutritional value. Both Figs 11 and 12 provides conclusive proof as to the fact that the stress variation during cell compression is non-linear. This behaviour agrees with the general stress-time variation discussed previously in this article.

**Fig 12:** Variation of stress with time during the cell compression simulation as affected by varying compression rates. (a) fresh cells (*X/X*_*0*_ = 1.0); (b) moderately dried cells (*X/X*_*0*_ = 0.5); (c) extremely dried cells (*X/X*_*0*_ = 0.1) (*X/X*_*0*_ is the normalised moisture content).

Fig 13 depicts the variation of strain with time during the cell compression simulation as affected by varying compression rates. Unlike the stress-time variation, strain-time variation reveals a linear behaviour. This is in alignment with the general strain-time variation discussed previously and commonly observed in all the dryness states. However, there is a pre-straining stage from 50 μs to approximately 70 μs, where the dried cells are compressed and initiates the next phase of rapid strain gaining through an initial force transmission.

**Fig 13:** Variation of strain with time during the cell compression simulation as affected by varying compression rates. (a) fresh cells (*X/X*_*0*_ = 1.0); (b) moderately dried cells (*X/X*_*0*_ = 0.5); (c) extremely dried cells (*X/X*_*0*_ = 0.1) (*X/X*_*0*_ is the normalised moisture content).

#### Force on the compression plate

Fig 14 shows the variation of force on the compression plate with time during cell compression simulation as affected by different turgor pressures. The force on the compression plate is the equal and opposite of the force on the cell applied by the compression plate. This force is a critical parameter for the design and implementation of machinery and processes for drying of fruits, vegetables and other biological materials. Accordingly, from Fig 14, it is evident that the force on the compression plate is the largest for fresh cells. For dried cells, the force is significantly lower compared to the fresh state. The implication of this observation is that the threshold force occurs during the compression of fresh cells. In other words, in terms of the stress-strain response, the cell or tissue is at its most sensitive or mechanically vulnerable at the fresh state. This can be a valuable insight for the food processing industry. For example, designing machinery or processes not to exceed the threshold stresses at fresh state would automatically ensure that the cell or tissue damage would not occur at other dryness levels.

The article "A three-dimensional (3-D) meshfree-based computational model to investigate stress-strain-time relationships of plant cells during drying" was published in 2020. Journal: PLoS One.

**Fig 14:** Variation of force on the compression plate with time during the cell compression simulation as affected by different turgor pressures. (a) fresh cells (*X/X*_*0*_ = 1.0); (b) moderately dried cells (*X/X*_*0*_ = 0.5); (c) extremely dried cells (*X/X*_*0*_ = 0.1) (*X/X*_*0*_ is the normalised moisture content).

Sensitivity towards cell wall properties. *Cell wall compression modulus (G)*. In Fig 15, the stress-strain relationships at varying values of cell wall compressive modulus (*G = E/3*, *where E is the Young’s modulus of the cell wall*) and different dryness levels have been presented. Here, the SPH-CG model predictions as well as comparable experimental findings [45] for different cell compression stages have been presented. As seen in Fig 15, the micromechanical behaviour of the SPH-CG cell model seems to be relatively unaffected by the varying *G* values even after reducing the typical *G* value by a factor of 100 (i.e. *G* = 18.00 MPa against *G* = 0.18 MPa). This is exemplified by virtually overlapping stress-strain curves corresponding to different values of *G* (as *G* is a representation of the cell wall stiffness). This condition seems to prevail at fresh conditions (Fig 15(a)) as well as moderately dried (Fig 15(b)) and extremely dried conditions (Fig 15(c)). At the same time, model predictions for cell micromechanical response seems to be significantly deviating from the experimentally observed behaviour [45] at all *G* values as seen from Fig 15. However, the degree of this discrepancy is relatively higher at fresh conditions and become less severe for the dried conditions as shown in the figure.

The article "A three-dimensional (3-D) meshfree-based computational model to investigate stress-strain-time relationships of plant cells during drying" was published in 2020. Journal: PLoS One.

**Fig 15:** The stress-strain relationship of cells as affected by different cell wall compressive modulus (*G*) values. (a) fresh cells (*X/X*_*0*_ = 1.0); (b) moderately dried cells (*X/X*_*0*_ = 0.5); (c) extremely dried cells (*X/X*_*0*_ = 0.1) (*X/X*_*0*_ is the normalised moisture content).

*Cell wall thickness (t)*. In Fig 16, the stress-strain relationships at varying values of cell wall thickness (*t*) and different dryness levels have been presented, along with related experimental findings [45, 46]. The micromechanical behaviour of the 3-D SPH-CG cell model seems to be sensitive to the cell wall thickness. However, the degree of sensitivity seems to be less intense. For instance, the stress-strain curves corresponding to cell wall thickness values in the range 0.1 ≤ *t* ≤ 12 μm do not show significant deviations compared to each other as observed from Fig 16(a), 16(b) and 16(c). When the *t* value is changed significantly to 100 μm, there seems to be a significant change in the stress-strain response. In addition, the model predictions for cell micromechanical response seems to have a discrepancy relative to the experimentally observed behaviour [45] at all *t* values as seen from the graphs in Fig 16. Again, the absence of cell-cell interactions and intercellular spaces could be the main cause for this.

**Fig 16:** The stress-strain relationship of cells as affected by different cell wall thickness (*t*) values. (a) fresh cells (*X/X*_*0*_ = 1.0); (b) moderately dried cells (*X/X*_*0*_ = 0.5); (c) extremely dried cells (*X/X*_*0*_ = 0.1) (*X/X*_*0*_ is the normalised moisture content).

#### Sensitivity towards cell size

To observe the effects of cell dimensions on the micromechanical behaviour, a cell with different dimensions was modelled using the same 3-D SPH-CG modelling approach. The larger cell was spherical in shape with a diameter of 200 μm while a typical cell diameter of 150 μm was used for all the previous simulations. Apart from the cell size and the subsequent particle numbers used to create particle geometries, all the other physicochemical parameters for the large cell were similar to those of the generic-sized cell as given in Table 3. In developing the corresponding particle-geometry for the larger cell, 2516 wall particles and 3708 fluid particles were used. Fig 17 contains a visual comparison of two cells of different sizes going through compression at various levels of dryness while Fig 18 has a graphical representation of the stress-strain relationships for the cells of different sizes going through compression.

**Fig 17:** SPH-CG model predictions for compression of dried cells of different cell sizes. (a) smaller cell (generic) (*D* = 150 μm); (b) larger cell (*D* = 200 μm); (*D* is the cell diameter and *X/X*_*0*_ is the normalised moisture content).

The article "A three-dimensional (3-D) meshfree-based computational model to investigate stress-strain-time relationships of plant cells during drying" was published in 2020. Journal: PLoS One.

**Fig 18:** The stress-strain relationship of cells as affected by different cell sizes. (a) fresh cells (*X/X*_*0*_ = 1.0); (b) moderately dried cells (*X/X*_*0*_ = 0.5); (c) extremely dried cells (*X/X*_*0*_ = 0.1) (*D* is the cell diameter and *X/X*_*0*_ is the normalised moisture content).

Fig 17 indicates that the qualitative nature of cell shrinkage and morphological response for the larger cell is approximately similar to that of the generic-sized cell. The quantitative information provided through Fig 18 provides further verification for this. The stress-strain relationship demonstrated through the curves in Fig 18(a), 18(b) and 18(c), seem to be closely aligned in general for the two cell sizes. However, at initial stages of the compression process, there seems to be slight discrepancies particularly for the fresh cell state (Fig 18(a)) and the moderately dried state (Fig 18(b)). This discrepancy is particularly noticeable at the low stress-strain values. One of the reasons behind this could be the inertial effects arising during the compression process of the larger cells.

## Conclusions

### A multipurpose flexible meshfree-based computational model

The meshfree-based computational model proposed in this article has conclusively demonstrated that it can favourably simulate stress-strain-time behaviour of dried plant cells that are being compressed. To the best of authors’ knowledge, this is the first computational study to model the micromechanical behaviour of plant cells that are being dried and compressed. In doing so, a three-dimensional (3-D) coupled Smoothed Particle Hydrodynamics and Coarse-Grained (SPH-CG) approach has been employed. The performance of the developed model has been evaluated under different biological and physical circumstances such as varying turgor pressures, strain rates, mechanical properties and cell sizes. Further, it has been pointed out that this meshfree-based computational model can be used to derive insights that are valuable in designing and implementing machinery and processes for plant biological materials (e.g. design of machinery for food drying processes). The fundamental computational framework of this modelling approach facilitates effective and flexible modelling of multiphase interactions and large deformations present in the plant cellular structure. Even though parenchyma cells have been used in this investigation as a representative plant cell category, the computational framework has clear capabilities in modelling other plant cell types. Furthermore, it has the potential and flexibility to move beyond the plant cells and simulate equivalent biological structures and processes such as dehydration and mechanical loading of animal cells.

The article "A three-dimensional (3-D) meshfree-based computational model to investigate stress-strain-time relationships of plant cells during drying" was published in 2020. Journal: PLoS One.

### Limitations of the proposed computational modelling approach

Although the SPH-CG computational modelling approach discussed in this article has demonstrated realistic capabilities in simulating the micromechanical response of dried plant cells that are being compressed, it can be observed that there are a few limitations of its performance when it comes to predicting the true micromechanical behaviour. For instance, at high strains, the model predictions for stress response deviates considerably from the experimentally observed behaviour. A key factor causing this behaviour is the absence of intercellular interactions in this single cell modelling approach used in this investigation. In the true plant cellular structure, the interactions from neighbouring cells as well as intercellular spaces have significant effects on the micromechanical as well as morphological response of a cell [1]. An oversimplification of the current modelling approach is using homogeneous properties for cell fluid and wall. In reality, there are variations of such properties (e.g. cell wall shear modulus, thickness and fluid properties) even across one single cell. In addition, the absence of cell wall plastic deformation can be given as a current limitation of the proposed computational modelling approach.

### Further potential extensions of the model

An immediately possible further extension of this 3-D SPH-CG computational modelling approach would be to embed heterogeneous properties such as heterogeneous cell wall and fluid properties into the model. This would facilitate closer approximations of real micromechanical behaviour seen through experiments. Another potential enhancement of the proposed computational cell model would be to incorporate plastic behaviour into the cell wall mechanical description which can be a promising endeavour based on current evidence. In addition, meshfree-based computational modelling approaches have previously been successfully used to model cell aggregates [18]. Therefore, modelling multi-cellular systems with embedded cell-cell interactions while taking intercellular spaces into account could enable better predictions. Based on previous evidence as well as the results presented in this article, it can be deduced that this computational framework can be applied to model micromechanics of small and large scale multi-cellular structures. Such applications could then be further extended to develop multiscale or bulk scale models, revealing mechanisms applicable to real biological materials and processes [48, 49]. By considering the nature of the proposed computational modelling approach, there are no fundamental difficulties in adopting the model to replicate other types of cells and complex micromechanical behaviours under different and extreme loading conditions. Since the meshfree-based SPH-CG models can inherently handle multiphase interactions, there can be numerous future applications of this model in different fields of engineering and biological sciences.

The article "A three-dimensional (3-D) meshfree-based computational model to investigate stress-strain-time relationships of plant cells during drying" was published in 2020. Journal: PLoS One.

## Supporting information

S1 File Quantitative data behind reported results in the article. (XLSX)

S2 File Simulation sample data outputs. (ZIP)
